RETRACTED

# Analysis of the Correlation between Football Education Environment and Students' Psychology Health Based on Gauss Characteristics

**DOI:** 10.1155/2022/9429846

**Published:** 2022-09-25

**Authors:** Shu Qiao, Gaosong Huang

**Affiliations:** ^1^Liaoning Shihua University, Institute of Physical Education, Fushun 113001, China; ^2^Institute of Physical Education, University of Huanggang Normal University, Huanggang 438000, China

## Abstract

Campus football has become a core content of school physical education. Through football education, we can cultivate students' sound personality and promote students' all-round physical and mental development. At the same time, through psychological skills training methods, we can enrich the educational methods of football skills and provide theoretical reference for promoting educational reform. On the basis of Gaussian features, this paper combines the mixed Gaussian feature model to further describe the relationship between football education and students' psychology. At the same time, Apriori association rule algorithm in data mining is introduced, and Apriori algorithm is improved in parallel with Hadoop data processing platform. Several parallel association rule algorithms are emphatically studied and analyzed to strengthen the analysis of the relationship between football education and students' psychology. The results show that the average recognition rate of the correlation between football education and students' psychology based on Gaussian features is 17.91% higher than that of ordinary results, which obviously improves the correlation recognition result and has a good descriptive ability. Therefore, it has become an important issue for today's physical education workers to analyze the correlation between football education and students' psychology in order to cultivate students' sports and mental health.

## 1. Introduction

At present, the social competition is fierce, the society is full of opportunities and challenges, and various factors such as employment difficulties also aggravate students' unhealthy psychological phenomena and mental disorders [1]. Students in school are the key growth stage of physiology and psychology, and some unhealthy activities fetter students' physical and mental health, career and self-realization, which also hinders the harmonious development of society [2]. Therefore, colleges and universities need to strengthen students' physical education, especially how college football education can promote students' mental health, and how to implement specific college football education activities. The construction of college football culture system can have a positive impact on students' psychological state. Through the organization and development of football education activities in colleges and universities, not only can students' psychological pressure in learning be transferred and alleviated but also a relaxed communication environment can be obtained, and the potential psychological burden can be fully released through physical exercises and exchanges of physical skills during their participation in football activities [3]. Therefore, college football education is a more effective way to promote students' mental health. At the same time, psychological skill training is also an important part of sports training, which is widely used in various sports training [4]. Practice has proved that psychological skill training can effectively help athletes get good training results in sports training. Therefore, applying psychological skills training to campus football teaching will definitely help students learn football skills efficiently.

RETRACTED

Because of its simplified rules, various forms and football games, football education has become a favorite sport for many students [5]. At the same time, football is also a sport that closely combines individuals and groups. It requires the unity, cooperation and joint efforts of peers, cultivates students' personal spirit of never giving up in the face of difficulties, courage to overcome difficulties and solve problems, and promotes the team spirit and cooperative consciousness of mutual trust, mutual understanding and cooperation among students, hons their perseverance in overcoming difficulties, cultivates their healthy psychological quality, strengthens their team consciousness, and lays a foundation for shaping students' perfect personality [6]. Therefore, football education activities are widely carried out in colleges and universities. At the same time, psychological education is an important part of cultural education. Implementing psychological education for students is the demand of comprehensively promoting the quality education of student athletes, training and bringing up high-quality laborers and outstanding sports reserve talents for the country, which is in line with the demand of healthy growth and all-round development of student athletes and the development trend of modern competitive sports [7]. However, the current cultural education does not pay enough attention to the psychological education of student athletes, and there is a lack of psychological education model for student athletes to guide practice. Building a fairly comprehensive and systematic psychological education model that is targeted at student sports groups and fully incorporated into the training system of “combination of sports and education” is therefore extremely important from a practical standpoint. Thus, there is a positive and mutually reinforcing relationship between football instruction and student psychology. This paper develops a set of research methodologies appropriate for analysing the relationship between college football education and students' psychology in order to demonstrate this argument. The mixed Gaussian feature model is combined on the basis of Gaussian characteristics to further describe the relationship between football education and students' psychology. Apriori association rule algorithm is introduced at the same time as Hadoop data processing platform, and Apriori algorithm is refined concurrently. In order to increase the examination of the relationship between football instruction and students' psychology, a number of parallel association rule algorithms are carefully examined and assessed.

RETRACTED

Gaussian feature uses Gaussian function as the basis to estimate the distribution of the signal at the bottom of the image, and its space is closely related to the Gaussian function space. Spatial function can better study and analyze the relationship between football education and students' psychology. Association rule mining is one of the most famous data mining methods [8]. Its main significance lies in finding out the hidden relationships among different items in the database, and the core problem is the acquisition of frequent item sets. From the initial application analysis to the present, it can be used in almost all kinds of fields that need to discover the laws between variables. The innovation of this paper lies in:

1. The Gaussian feature is associated with mathematics, which is proposed based on the fact that the covariance feature lacks the mean information and cannot form a complete Gaussian estimate. It not only contains the mean information but also has the ability of describing spatial information by probability density function. Therefore, Gaussian feature is introduced to describe the relationship between football education and students' psychology in order to improve the whole recognition rate
2. Improvements to the Apriori association rule algorithm through parallelization include fewer cyclic calls during operation, faster startup, and increased algorithmic effectiveness. The notion of figuring out the highest order is advanced. Prior to mining frequent item sets, it is possible to narrow down the candidate item set pool and save network traffic by identifying the highest order of potential frequent item sets

## 2. Related Work

The education of college students seeks the breakthrough point of quality education in the balance between mental health and physical education, in order to gradually improve the educational content [9]. The object of quality education must face all students, and strive to cultivate students into all-round talents. Therefore, the requirements of students' physical and mental development should reach a harmonious height [10]. The education of mental health needs to start from the students' own psychological and physiological conditions, and improve their psychological quality through psychological education. At the same time, scientific and reasonable educational methods must be applied in physical education, so that students can be familiar with and master the skills of coordinated development of health care and physical fitness, strengthen their physique, and cultivate their sports ability, so as to develop quality-oriented educational activities in an all-round way.

RETRACTED

Bozkurt et al. put forward that according to the medical examination data, according to their health status, physical strength and cardiovascular function, combined with their individual characteristics such as living environment and sports hobbies, appropriate exercise types, time and frequency should be prescribed in the form of prescription, and points out matters needing attention in exercise, so as to carry out regular exercise in a planned way to achieve the purpose of fitness or treatment, that is, exercise prescription [11]. Zhang and Hongxin's task to participate in football can cultivate the students' willpower, such as hard work and enterprising, unity and cooperation, tenacity and courage. Therefore, football can promote the mental health cultivation of teenagers and the shaping of their willpower [12]. Li thinks that the development of campus football should give play to the educational function of football, promote the popularization of campus football and promote the common development of culture and skills [13]. Wang thinks that the teaching and training process of campus football cannot be across the board like the traditional method, but should carry out appropriate teaching and training contents according to the characteristics of teenagers' physical and mental development, and formulate corresponding strategic contents suitable for students' physical and mental development according to the characteristics of different stages [14]. Stambulova and Johnson believe that the educational nature of campus football means not only teaching students sports knowledge and skills but also integrating knowledge of other disciplines into it, and carrying out health education from the perspective of mental health and social adaptation, so as to improve students' sports quality and psychological level of physical activities [15]. According to Bai, a psychological quality that is internally created by the interaction of genetics and environment is what constitutes mental health. This quality is rather constant. These psychological traits influence or determine an individual's psychological, physiological, and social functions, which in turn influence the status of the individual's mental health [16]. Tryon thinks that psychological quality refers to the ability of human body in psychological activities, that is, the comprehensive ability to cope with, undertake and resolve all kinds of cardiogenic stress, and it is mainly manifested in emotional and behavioral tendencies [17]. Codreanu et al. think that psychological quality is a kind of ability to integrate the contradiction between individual self-satisfaction and social expectation, which is shaped by the combination of heredity and environment, and it is a balance ability to adjust the conflict between expectation and realistic ability [18]. Kipp et al. established the first sports psychology laboratory in the world, and the research of sports psychology began to get on the right track [19]. Chraif and Dumitru pointed out that the characteristics of sports psychology workers' topic selection are as follows: psychological training research serving sports teams to improve sports performance is in a leading position, and sports teaching research has obviously increased, which fully reflects the clear research orientation and important application value of sports psychology [20].

RETRACTED

Students' physical and mental development as well as their cognition, consciousness and emotion are mutually coordinated and supportive. Apart from knowledge education, students should cultivate healthy personality. While developing students' sports achievements, they should pay more attention to their inner thoughts and true feelings. This is the core task and value embodiment of quality education. In the classroom education, students' development should be taken as the starting point, the teaching contents of psychology and physical education should be perfectly combined, football education activities should be fully tapped, and a good psychological state should be cultivated in the exercise of activities to help students grow healthily. In addition, in terms of physical education, we should also change from primitive physical education to cultural education in a broad sense. Instead of simply carrying out physical education, we should impart physical skills and knowledge to students, constantly strengthen their physique, so as to achieve the goal of all-round development. We should pay close attention to the cultivation of students' psychological quality, make students develop good physical exercise habits, cultivate healthy lifestyles and behaviors, and realize the coordinated development of their whole body and mind. Therefore, we must make efforts to enrich and improve education and integrate mental health education content.

RETRACTED

## 3. Methods

### 3.1. Gaussian Mixture Feature Model

Covariance feature is currently the superior way for feature description. A channel signal's covariance matrix is a matrix, but due to its symmetry, it has a far smaller actual dimension than the histogram's, which grows exponentially as more channels are added [21]. Additionally, covariance can be utilised to combine many attribute features. Various covariance matrices result in curves or surfaces that represent various signals. In order to generate a complete Gaussian estimate, covariance characteristics need the mean information, which they lack. In addition to the mean information, it can also describe the spatial information of the probability density function.  Figure 1 depicts the characteristics of its spatial distribution.

According to the Gaussian spatial distribution diagram, covariance is not a Gaussian distribution of complete parameters, and it lacks important mean vector parameters. If the Gaussian distribution of complete parameters is used to estimate the signal probability density function characteristics of a signal, a more comprehensive and accurate feature descriptor can be obtained than the regional covariance, and an effective feature correlation analysis can be made for football education and students' psychological characteristics.

Gaussian distribution is determined by the mean vector *μ* and covariance matrix ∑[], and its corresponding signal probability density function features are called Gaussian features, which are expressed as follows:

(1) $$\begin{array}{c} M=\left[P_{1}^{\mu }\right], \end{array}$$

where *M* is the positive definite lower triangular affine transformation matrix, *μ* is the mean value of Gaussian distribution, and *P* is the positive definite lower triangular matrix obtained by decomposing the covariance matrix ∑[] of Gaussian distribution. Because the covariance matrix is a positive definite symmetric matrix, the factorization result must exist, and if the *P* matrix is defined as a positive definite lower triangular matrix, *P* can be obtained uniquely. Such *P* transformation *Z* = *PZ*_0_ + *μ* is called positive definite lower triangular affine transformation, and the corresponding matrix transformation expression is as follows:

(2) $$\begin{array}{c} \left[Z\right]=M*\left[Z_{0}\right]={PZ}_{0}+\mu . \end{array}$$

To sum up, the associated positive definite lower triangular affine transformation matrix *M* can transform any Gaussian distribution into a standard Gaussian distribution. Therefore, the corresponding *M* can represent the corresponding Gaussian distribution.

RETRACTED

A feature is equivalent to a corresponding multidimensional Gaussian distribution, which is a single Gaussian model that is often applied in the field of multimedia processing. However, from the meaning of probability density function of single Gaussian distribution, it can be known that two-dimensional points obeying single Gaussian distribution should be approximately elliptical on the plane; a three-dimensional point that obeys a single Gaussian distribution should be approximately ellipsoidal in space. Then, some data distributions cannot be accurately described by single Gaussian distribution. When there is a pile of sample data that does not present an ellipse on a two-dimensional plane, the effect of single Gaussian modeling is definitely not good, so we should consider using another strong descriptive model that has been affirmed in the field of multimedia-mixed Gaussian feature model to describe it. The strong descriptive power of Gaussian mixture feature model is shown in Table 1.

The Gaussian mixture feature model is composed of the weighted sum of several single Gaussian models. It can be seen from the table that the description, probability distribution, and weighting coefficient of the mixed Gaussian feature model are stronger and more effective than those of the single Gaussian model, and it is more suitable for the analysis of the relationship between football education and students' psychology. When the number of models is properly selected and the sample set is sufficient, it is enough to approximate any distribution with any accuracy.

Mathematically, the probability density function of the Gaussian mixture feature model is defined as follows:

(3) $$\begin{array}{c} p\left(x_{i}\right)=\overset{M}{\underset{j=1}{\sum }}\alpha_{j}N_{j}\left(x_{j},\mu_{j},\underset{j}{\sum }\right), \end{array}$$

where *x*_*i*_ is any random vector {*x*_*i*_|1 ≤ *i* ≤ *N*|}, *α*_*j*_ is the weighting coefficient, and *M* is the number of Gaussian models. The calculation method of each *N*_*j*_(*x*_*j*_, *μ*_*j*_, ∑_*j*_) is shown in Equation (3), which represents the *M*th Gaussian distribution.

Estimate the Gaussian distribution of each sample point under each model by Equation (4):

(4) $$\begin{array}{c} \beta_{ij}=E\frac{\alpha_{j}N_{j}\left(x_{i}\right)}{\sum_{1}^{M}\alpha_{i}N\left(x_{i}\right)}. \end{array}$$

See Equations (5), (6), and (7) for the update of each parameter *α*_*j*_, *μ*_*j*_, and ∑_*j*_:

(5) $$\begin{array}{c} \alpha_{j}=\frac{\sum_{i=1}^{N}\beta_{ij}}{N}, \end{array}$$

(6) $$\begin{array}{c} \mu_{j}=\frac{\sum_{i=1}^{N}\beta_{ij}x_{i}}{\sum_{i=1}^{N}\beta_{ij}}, \end{array}$$

(7) $$\begin{array}{c} \underset{j}{\sum }=\frac{\sum_{i=1}^{N}\beta_{ij}\left(x_{i}-\mu_{j}\right)}{\sum_{i=1}^{N}\beta_{ij}}. \end{array}$$

When the condition *i* = 1 is met, it ends. Generally, *μ* = 10.5 is obtained by Equation (7), and ∑_*j*_ is obtained after the step; that is, the iteration ends when the parameter is updated to be almost unchanged.

RETRACTED

### 3.2. Apriori Association Rule Algorithm

As an important part of the field of data mining, association rules can quickly and effectively find the existing, hidden and valuable association relationships among various transaction items from the specified data sets, so as to provide powerful decision support for users. Therefore, association rules can effectively mine the valuable association between football education and students' psychology. The creation of frequent item sets and the creation of powerful association rules are the two main components of traditional association rules mining. Apriori association rules algorithms include breadth-first search algorithm, depth-first search algorithm, data set division algorithm, sampling algorithm, incremental updating algorithm, etc., according to various standards. It is possible to sum up the generation of association rules as the generation of frequent item sets and the generation of powerful association rules. The foundation for the subsequent calculation is the initial step. In order to assess the effectiveness of the association rules algorithm, it is crucial to frequently construct item sets. Users must establish a minimum support threshold and a minimum confidence threshold during operation to prevent the creation of a large number of frequently occurring item sets and association rules.  Figure 2 depicts how the Apriori association rule algorithm functions.

Apriori algorithm has two characteristics in the process of operation: first, the algorithm needs to calculate layer by layer and repeat operations. All possible candidate item sets are generated by connecting the frequent item sets obtained in the first operation, and the frequent item sets are obtained after traversing the transaction sets. Next, the final item sets are obtained from the frequent item sets by using the same method, and the frequent final item sets are obtained by cyclic operations. The formula for connection is as follows:

(8) $$\begin{array}{c} Ck=L_{k-1}00L_{K-1},\\ Ck=\left\{A00B\left|A,B\in L_{k-1},\right|A\cap B=k-2\right\},\\ Ck=\alpha 00\beta *L_{k-1}. \end{array}$$

Secondly, the pruning strategy is used in the process of generating candidate item sets, and the frequent items calculated in the last round are used. When connecting sets to generate high-order candidate sets, the newly obtained candidate sets are reduced by prior properties. Then, by counting the support count of each candidate item set, and comparing with the given minimum support count, the candidate item set whose support count is greater than the given threshold is output.

RETRACTED

The algorithm is parallelized completely according to the operation process of Apriori algorithm. Because the iterative operation layer by layer runs on Hadoop platform, the efficiency of the algorithm is greatly improved compared with the original Apriori algorithm, and the memory overhead can be effectively reduced. Combining with Hadoop data processing platform, the Apriori algorithm is parallelized and improved. The running process of Hadoop data processing platform is shown in Figure 3.

The reliability of Apriori association rule calculation is provided by the reliability of Hadoop architecture. Hadoop can automatically maintain multiple copies of data and automatically redeploy the calculation task after the task fails, which can ensure that the node failure will not lead to the calculation failure, so it is suitable for discovering the correlation between football education and students' psychology.

In order to better evaluate the performance of Hadoop data processing platform, we use Java to write a multithreaded program as the traditional parallel association rule program (the reason for using Java is that the parallel association rule program based on Hadoop is also implemented in Java, so it can be better compared by using the same language). The main thread of Java multithreaded program reads the file and distributes the data and candidate set information to *N* threads. *N* corresponds to the setting of map capabilities, which are 2, 4, 8, and 16, respectively, as shown in Table 2.

From the results in Table 2, after parallelizing Apriori algorithm combined with Hadoop data processing platform, the map capability is larger and the data set is larger. The performance of Hadoop-based parallel association rule program is obviously better than that of Java multithread association rule program, but with the expansion of data set, the gap is getting bigger and bigger. Therefore, combining Hadoop data processing platform to parallelize Apriori algorithm can improve the performance of association rule analysis algorithm, which is helpful to further analyze the relationship between football education and students' psychology.

RETRACTED

## 4. Experimental Analysis

Given the distinct application domains of football instruction and student psychology, a Gaussian feature can reduce the impact of individual characteristics on mental health and enhance discriminating between the two types of features. With unknown samples, it is extremely practical and compatible. The capacity of various features to describe themselves when biassed is the main focus of the first analysis. Comparison of the result curve is necessary to determine whether Gaussian features can increase the effectiveness of mental health identification. The curve representing the result under the Gaussian feature is shown in Figures 4 and 5. Each outcome curve depicts the degree to which the connection between student psychology and football education is recognised.

By comparing the two result curves, it can be seen that the average recognition rate of the correlation between football education and students' psychology based on Gaussian features is 17.91% higher than that of ordinary results, which obviously improves the correlation recognition result, has a good descriptive ability, and can get the following correlation analysis conclusions.

Students in the experimental group participating in campus football activities have better ability to adapt to the environment and physical and mental changes in their daily study and life. The experimental group students have better interpersonal quality and ability. The students in the experimental group showed a strong sense of adventure and independence in their study and life, a strong willpower, and a strong sense of responsibility in the process of achieving their goals, and they were able to cope with setbacks well, and they were more receptive and inclusive to people and things around them. The experimental group students have a positive understanding of self-cognition. The experimental group students can adopt various coping strategies and methods to deal with the problems they face and their related emotional troubles. In the campus football education, psychological skill training which accords with the characteristics of youth football learning is added, and two commonly used methods of mental skill training, namely, representation training and suggestion training, are combined and matched, and then infiltrated into football education to help students learn football technical knowledge. It is found that experimental psychological skills training can help students master football skills faster and more accurately in campus football education, so as to improve students' learning efficiency. Therefore, the relationship between football education and students' psychology is complementary and mutually reinforcing.

RETRACTED

In the field of object detection, evaluating the performance of an algorithm is mainly to evaluate the analytical performance of its corresponding model, and the evaluation of model quality is mainly measured by the mixed Gaussian characteristic curve. Specifically, this paper is to evaluate the performance of the built model by the mixed Gaussian characteristic curve. The Gaussian mixture characteristic curve is shown in Figure 6.

As can be seen from Figure 6, the corresponding Gaussian mixture characteristic curve based on the model can be obtained, and the performance of the model can be directly reflected by the Gaussian mixture characteristic curve. Usually, when the model is evaluated, it is required to maintain a low false detection rate when it reaches a certain false detection rate. Therefore, it can be seen from the curve shown in Figure 6 that the false detection rate of the mixed Gaussian curve tends to 0.129 when the iteration basically ends, which indicates that the performance of the mixed Gaussian feature model is excellent, and it is suitable for analyzing the relationship between football education and students.

The minimum support and minimum credibility of Apriori association rule algorithm proposed in this paper can be changed at any time, which greatly facilitates the needs of users. The improved Apriori association rule algorithm mining object is very clear, which improves the mining efficiency and reduces the space complexity. The improved Apriori association rule algorithm only scans the database once, which greatly improves the running efficiency of the algorithm and reduces the time complexity. The above algorithm is tested in the same environment, and the specific test results are shown in Figure 7.

This paper offers a very in-depth analysis of the Apriori association rule algorithm's concept and method. In order to learn more about the Apriori algorithm, a test is used to illustrate how it works and its flaws are examined. This work describes the basic implementation processes of the improved algorithm, provides an experimental comparison between the new algorithm and the existing algorithm, and to some extent improves the Apriori association rule algorithm based on the shortcomings of the existing algorithm. The experimental results demonstrate that the revised algorithm runs substantially faster than the Apriori approach when the minimal support is relatively low. The technique takes about the same amount of time to run when the minimum support gradually increases; however, the improved approach takes a lot less time than the Apriori algorithm to run when the number of transactions is growing. The final test results demonstrate that the revised algorithm performs significantly better than the original algorithm in terms of both performance and efficiency.

RETRACTED

In order to analyze the details of the performance of Hadoop-based parallel association rules program, we counted the start running time and duration of each association rule in Hadoop, and counted the start running time and duration of each internal stage of each association rule, as shown in Figure 8.

Hadoop architecture is not started until a map is found. In this experiment, the map was completed 15 s or 20 s after the MAP was completed. As both setup and cleanup take at least 2 s, reduce also takes more 8 s or 11 s. If the execution time of the map phase is too short, the analysis using Hadoop is obviously slower than the common Java multithreading program. For the analysis of very large-scale data sets, the execution time of map phase will take up the main part of the whole calculation time, which is slightly slower than Java multithreading program in theory. On the premise of multiple computing nodes, the Java multithreading program can achieve the purpose of parallelism through socket. For the convenience of discussion, this program is called Java-socket multithreading program. Due to the lack of the support of file system like HDFS, the data of Java-socket program comes from one node. Common clusters are generally connected by Gigabit Ethernet. The number of nodes in the cluster is set at 30, and each node is equipped with 1500 association rules. From our experiment, it can be seen that the time for each core to process a file is about 2 s, which is equivalent to processing 15 M of data in 1 s. For Java-socket multithreaded programs, due to the limitation of IO, the processing speed cannot reach the cumulative effect, and it can only reach more than 100 m at most. Parallel rule program based on Hadoop, supported by HDFS file system, the data of each computing node basically comes from its own node or neighboring nodes, which is not limited by IO, and the processing speed can achieve the effect of accumulation on the premise of very large data set. Therefore, the Hadoop-based parallel association rules program is suitable for processing very large data sets.

## 5. Conclusions

Based on the relationship between football education and students' psychology, this study verifies the effect of the combination of psychological skills training methods in football technology education, enriches the educational methods of football technology, and provides theoretical reference for promoting educational reform. In order to improve students' learning efficiency in campus football education, it is an inevitable trend of educational development to introduce advanced educational methods. Only by breaking the stereotypes and boldly innovating can good educational effects be achieved. Introducing psychological training into football education classroom can enrich the means and methods of football education on campus. Establishing a relatively complete school-based football education and training system can improve students' learning efficiency and solve the difficulties and problems encountered by students in education and training. At the same time, it provides a novel method of football training in education, which can improve the multiangle and diversification of students' learning efficiency.

RETRACTED

In this paper, based on Gaussian features, the correlation features of football sports education and students' psychology are extracted, respectively. Through the mathematical analysis of the existing common single sports features, it is found that they are basically composed of the average of each joint movement information. Combined with the Gaussian features based on covariance features, the Gaussian features of each sample are extracted for subsequent recognition rate experiments. Then, through the extraction of Gaussian mixture features, the Gaussian mixture model can obviously have better advantages: strong adaptability and robustness. Therefore, on the basis of Gaussian features, mixed Gaussian features are introduced in order to achieve a comprehensive description of different categories of relevance. At the same time, based on the analysis of existing parallel association rule algorithms, Apriori association rule algorithm based on Hadoop is proposed. The main difference between Apriori association rules algorithm based on Hadoop and traditional algorithms is that the introduction of candidate sets and the acquisition of frequent item sets only run once in the main process. Hadoop is a platform with good fault tolerance, so the program implemented by Hadoop-based parallel association rules algorithm can be executed when some nodes fail. Compared with the traditional parallel association rule algorithm, the data of Hadoop-based parallel association rule algorithm is not divided once at the beginning, but distributed in batches according to the capacity of each node for calculation, so the dynamic balance problem of the cluster can also be solved.

In this paper, the relationship between football education and students' psychology is studied, and the experiment is analyzed by Gaussian features. The function of Apriori association rules algorithm is also applied at the primary level, but there are still many problems that need to be improved in the next step. For Apriori association rule algorithm, although the running efficiency has been improved, it will still generate a large number of candidate item sets when generating data, which will increase the traffic between networks, especially when running on dense data sets. In the next step, we will continue to look for pruning strategies to further reduce the network traffic. The problem of selecting the number of models with Gaussian mixture features needs to be deeply analyzed in combination with data sets. Whether the number of models is appropriate or not largely determines the strength of feature description. How to give an objective and fair number selection mechanism is also a problem worth studying in the follow-up work.

RETRACTED

## Figures and Tables

**Figure 1:** Spatial distribution characteristic diagram.

**Figure 2:** Operation process of Apriori association rules.

**Figure 3:** Operation process of Hadoop data processing platform.

**Figure 4:** Correlation curve.

**Figure 5:** Recognition rate curve.

**Figure 6:** Gaussian mixture characteristic curve.

**Figure 7:** Test results.

**Figure 8:** Improved parallel association rules of Hadoop.

**Table 1:** Strong descriptive power of Gaussian mixture feature model.

Different types	Strong descriptive power	Probability distribution	Weight number
Single Gaussian model	89.142	0.885	1.782
Gaussian mixture feature model	97.873	0.937	1.994

**Table 2:** Performance evaluation table of Hadoop data processing platform.

Data set	Calculate the running time when the number of threads is 2	Calculate the running time when the number of threads is 4	Calculate the running time when the number of threads is 8	Calculate the running time when the number of threads is 16
A	85 s	54 s	39 s	31 s
B	153 s	88 s	52 s	41 s
C	358 s	145 s	85 s	73 s

## Data Availability

The data used to support the findings of this study are available from the corresponding author upon request.
